The article "Analysis of Continuous Nursing Intervention on Aplastic Anemia Patients Based on the “Information-Motivation-Behavioral Skills Model”" was retracted in 2023. Reasons: unreliable results or conclusions; concerns about the data; concerns about the peer review; concerns about the citations.

# Analysis of Continuous Nursing Intervention on Aplastic Anemia Patients Based on the “Information-Motivation-Behavioral Skills Model”

**DOI:** 10.1155/2021/8204522

**Published:** 2021-10-18

**Authors:** Wei Shen, Xiaorong Liu, Aiping Zhou

**Affiliations:** Department of Hematology, The First Affiliated Hospital of Soochow University, SuZhou, Jiangsu 215006, China

## Abstract

**Objective:**

To explore the effect of continuous nursing care based on the “information-motivation-behavioral skills model” (IMB) in the intervention of patients with aplastic anemia.

**Methods:**

A total of 90 patients with aplastic anemia who were admitted to our hospital from June 2019 to January 2021 were included in the study. The patients were divided into an observation group and a control group according to the random number table, with 45 patients in each group. The control group received routine nursing care, while the observation group received continuous nursing care based on IMB on the basis of the control group. Patients were followed up for 3 months, and their health knowledge was assessed with our self-made health knowledge rating scale. Patients' medication compliance was assessed using the Morisky medication compliance questionnaire. The self-care ability was assessed with the self-made self-care ability scale in our hospital. The comprehensive quality of life assessment questionnaire (GQOLI-74) was used to assess the quality of life of patients. A self-prepared nursing satisfaction questionnaire was used to score patients' nursing satisfaction. The total effective rate of nursing was evaluated.

**Results:**

The awareness scores of basic disease knowledge, medication knowledge, and daily self-care knowledge in the observation group were higher than those in the control group (*P* < 0.05). The scores of medication compliance in the observation group were higher than those in the control group (*P* < 0.05). The self-care abilities such as healthy diet, psychological adjustment, self-care skills, oral care, and perianal care in the observation group were higher than those in the control group (*P* < 0.05). The quality of life scores of patients in the two groups in the 3 months of nursing were higher than those when they were discharged from hospital (*P* < 0.05). The GQOLI-74 score of 3 months' nursing care in the observation group was higher than that in the control group (*P* < 0.05). The nursing satisfaction degree of the observation group (97.78%) was higher than that of the control group (82.23%) (*P* < 0.05). The total effective rate of nursing care in the observation group (97.78%) was higher than that in the control group (77.78%) (*P* < 0.05).

The article "Analysis of Continuous Nursing Intervention on Aplastic Anemia Patients Based on the “Information-Motivation-Behavioral Skills Model”" was retracted in 2023. Reasons: unreliable results or conclusions; concerns about the data; concerns about the peer review; concerns about the citations.

**Conclusion:**

IMB-based continuous nursing care can significantly increase the awareness of health knowledge in patients with aplastic anemia, effectively improve medication compliance, significantly enhance self-care ability, and thus, improve the quality of life.

## 1. Introduction

Aplastic anemia is a common disease in the blood system, and its inducing factors are relatively complicated. The exact etiology is not clear, which may be related to chemical poisons, viral infection, lack of immunity, and other factors. The clinical manifestations are low proliferation of bone marrow hematopoietic cells and peripheral blood pancytopenia, which are mainly anemia, hemorrhage, and infection. With the gradual progress of the disease course, the disease could be aggravated and seriously threaten the life and health of patients. At present, immunosuppressants such as cyclosporine are commonly used in the treatment of aplastic anemia in clinics. By improving the patients' hemorheological indexes, the patients' condition was significantly relieved. Aplastic anemia is prone to repeated attacks due to a long course of treatment. Discontinuation of medication and improper nursing can have an adverse effect on the clinical efficacy and even lead to worsening of the disease [1–3]. Relevant research shows that effective continuous care for patients with aplastic anemia after discharge can improve patients' medication compliance and enhance patients' self-care ability by providing targeted health guidance [4]. At present, continuous nursing based on the information-motivation-behavioral skills model (IMB) has become a personalized and targeted clinical nursing management mode. In this model, individual information and motivation can activate behavioral skills, which indirectly trigger the generation and maintenance of intervention behaviors. Nursing researchers can formulate intervention plans according to IMB to study the effects of nursing interventions on specific behaviors. As a behavior change model, the IMB model emphasizes the intervention of patients' information, motivation and behavior and promotes behavior change, which can enhance patients' awareness of self-care and ultimately achieve the goal of improving their quality of life [5–7]. However, there is little research on the application of this method in the intervention of aplastic anemia patients. This study used continuous nursing based on the IMB model to explore the effect of postdischarge intervention for patients with aplastic anemia. The report is as follows.

## 2. Data and Methods

### 2.1. Clinical Data

A total of 90 patients with aplastic anemia who were admitted to our hospital from June 2019 to January 2021 were selected as the research subjects. Inclusion criteria: (1) All patients met the diagnostic criteria of aplastic anemia. (2) First hospitalization, without receiving systematic health education. (3) Clear consciousness and have the ability of language communication. (4) The condition is basically stable. (5) Met the requirements of medical ethics, and the patients and their families signed informed consent. Exclusion criteria: (1) Complicated with heart, liver, kidney, and other important organ dysfunction. (2) Combined with cognitive or mental disorders such as senile dementia. (3) There are serious complications. (4) Withdrawal from the investigation midway for some reason. The patients were divided into an observation group and a control group according to the random number table, with 45 patients in each group. General patient data are presented in Table 1. There was no significant difference in general information between the two groups (*P* > 0.05).

The article "Analysis of Continuous Nursing Intervention on Aplastic Anemia Patients Based on the “Information-Motivation-Behavioral Skills Model”" was retracted in 2023. Reasons: unreliable results or conclusions; concerns about the data; concerns about the peer review; concerns about the citations.

### 2.2. Nursing Methods

The control group received routine nursing care; that is, hospital nurses gave discharge guidance according to the routine nursing care for patients with aplastic anemia. Before leaving the hospital, patients should be given health guidance on medication, diet, and cleaning of the mouth and anus. Review time was agreed, and love cards were issued, so that patients could contact the medical staff of the department at any time and ask questions about diseases. Telephone follow-up was conducted within the first week of discharge to answer patient's questions related to diseases. Telephone follow-up was conducted once a month after discharge, so as to know the rehabilitation of patient and the implementation of the doctor's advice and give the corresponding guidance. For patients with special needs, the number of telephone follow-up visits shall be increased according to the specific situation.

The observation group received continuous nursing based on IMB on the basis of the control group [8–10]. (1) Information intervention: nursing staff actively communicated with the patients, collected the specific conditions of the patients, mined and analyzed the information of the patients, summarized the needs of patient care and health education at discharge, and pushed the related health education knowledge based on the patients' needs through communication means such as WeChat and telephone, with the contents including introduction of aplastic anemia, the latest treatment progress, healthcare, prevention and control of complications, condition observation, psychological care, dietary care, and medication care. The content forms were as diverse as possible to improve the patients' reading interest. (2) Motivation intervention: patients with aplastic anemia require a long rehabilitation period. In addition to immunosuppressive drugs, bad living habits should be changed in the rehabilitation of patients. In the early stage of nursing, trust relationship was established with nurses to encourage caregivers to express their concerns and understand the real psychological state of caregivers. We should guide patients to realize the important significance of changing bad living habits and timely correct the negative feelings of patients' mental psychologically. According to the patients' medication rules, we should formulate scientific plans. Long-term administration of immunosuppressive drugs may damage the liver and kidney function of patients, so the medication plan should be reasonably adjusted in combination with the recent physiological data of patients and other indicators, to avoid adverse drug reactions and, thus, achieve a better therapeutic effect. The medication plan was evaluated every week, and the plan was fed back and corrected in time. If patients had any questions about medication, they could ask the medical staff through WeChat, etc., so that the problems could be effectively solved in the shortest time. (3) Behavioral skill intervention: research nurses' intervention on possible problems in the process of information intervention, routine nursing plan, and psychological rehabilitation plan was conducted through the WeChat group and telephone interview, and the related knowledge videos of caring for blood tumor patients were uploaded twice a week. The caregivers were followed up once a week to timely understand the physical condition of patients and effectively monitor their diet, medication, and other compliant behaviors. When necessary, they make a home visit.

The article "Analysis of Continuous Nursing Intervention on Aplastic Anemia Patients Based on the “Information-Motivation-Behavioral Skills Model”" was retracted in 2023. Reasons: unreliable results or conclusions; concerns about the data; concerns about the peer review; concerns about the citations.

### 2.3. Observation Indicators

1. The patients were followed up for 3 months and assessed with the self-made health knowledge rating scale in our hospital. The scale included three assessment items of disease basic knowledge, medication knowledge, and daily self-care knowledge, and the score range of each assessment item was 0–50 points. The higher the score was, the better the patients' health knowledge awareness would be. The total Cronbach *α* coefficient of the scale was 0.83.
2. Two groups were assessed for medication compliance using the Morisky medication compliance questionnaire, which consisted of eight items with a total of 8 points. Among them, the score <6 was classified as poor medication compliance, with the score between 6 and 7 as medium medication compliance and the score 8 as good medication compliance.
3. After a follow-up of three months, the self-care ability in healthy diet, psychological adjustment, self-care skills, oral care, and perianal care was assessed using the self-care ability scale developed by our hospital. The total Cronbach *α* coefficient of the scale was 0.74.
4. The comprehensive quality of life assessment questionnaire (GQOLI-74) was used to assess the quality of life of patients in the two groups at the time of discharge and 3 months of nursing care. The scale included four dimensions such as psychological function, social function, physical function, and material life, and the score for each dimension ranged from 0 to 100 points. The higher the score, the higher the quality of life of patients.
5. Nursing satisfaction was distributed to patients in the form of a self-prepared nursing satisfaction questionnaire for scoring. The satisfaction questionnaire included information intervention effect, motivation intervention effect, behavior skills intervention effect, nursing efficiency, nursing technology 5 aspects, and full scores of 100. Very satisfied: the score is above 80 points; satisfaction: the score ranged from 60 to 80; and unsatisfactory: the score was below 60 points. Nursing satisfaction = (satisfactory + relatively satisfactory)/total number of cases × 100%. The total Cronbach *α* coefficient of the scale was 0.81.
6. The total effective rate of nursing care was evaluated after follow-up for three months. The total effective rate of nursing included the following: marked effective: after nursing, the incidence of complications such as anemia and heart failure was significantly reduced, and the coordination degree of various treatments and nursing was good. Effective: after nursing, the incidence of complications such as anemia and heart failure was improved, and the coordination degree of various treatments and nursing was average. No effect: no improvement or aggravation of symptoms after care. Total effective rate of nursing = (number of cases with remarkable effect and effective effect)/total number of cases × 100%.

## 3. Statistical Methods

All data were analyzed by SPSS22.0 statistical software, and measurement data were expressed as mean standard deviation. An independent-sample *t* test was used for pairwise comparison. The count data were expressed as the rate (%) using the *χ*^2^ test. *P* < 0.05 indicated that the difference was statistically significant.

## 4. Results

### 4.1. Comparison of Health Knowledge Awareness between the Two Groups

The awareness scores of basic disease knowledge, medication knowledge, and daily self-care knowledge in the observation group were higher than those in the control group, and the difference was statistically significant (*P* < 0.05), as shown in Figure 1.

The article "Analysis of Continuous Nursing Intervention on Aplastic Anemia Patients Based on the “Information-Motivation-Behavioral Skills Model”" was retracted in 2023. Reasons: unreliable results or conclusions; concerns about the data; concerns about the peer review; concerns about the citations.

### 4.2. Comparison of Medication Compliance between the Two Groups

The scores of medication compliance in the observation group were higher than those in the control group, and the differences were statistically significant (*P* < 0.05), as shown in Figure 2.

### 4.3. Comparison of Self-Care Ability between the Two Groups

The self-care abilities such as healthy diet, psychological adjustment, self-care skills, oral care, and perianal care in the observation group were higher than those in the control group, and the differences were statistically significant (*P* < 0.05), as shown in Figure 3.

### 4.4. Comparison of Quality of Life between the Two Groups

There was no significant difference in the scores of psychological function, social function, physical function, and material life between the two groups at the time of discharge (*P* > 0.05). The QOL scores in the 3 months of nursing were higher than those when the patients were discharged from hospital (*P* < 0.05). The scores of QOL in 3 months of nursing of the observation group were higher than those of the control group, and the differences were statistically significant (*P* < 0.05), as shown in Figure 4.

### 4.5. Comparison of Nursing Satisfaction between the Two Groups

The nursing satisfaction degree of the observation group (97.78%) was higher than that of the control group (82.23%), and the differences were statistically significant (*P* < 0.05), as shown in Figure 5.

### 4.6. Comparison of the Total Effective Rates of Nursing Care between the Two Groups

The total effective rate of nursing care in the observation group (97.78%) was higher than that in the control group (77.78%), and the differences were statistically significant (*P* < 0.05), as shown in Figure 6.

## 5. Result

It is difficult to treat aplastic anemia clinically. Although clinical treatment can improve the prognosis of patients, the treatment cycle is long, and patients need to continue treatment after discharge. It should be noted that it is difficult for patients to obtain effective healthcare and guidance after discharge, which may affect the rehabilitation effect of the patients, leading to deterioration of their condition, and the patients have to be hospitalized again [11–13]. Therefore, patients with aplastic anemia still need continuous care after being discharged from hospital. Through implementing necessary diet, medication guidance, and health education, we can enhance our self-care management ability, improve patients' understanding of the disease, and narrow the doctor-patient relationship [14].

In this study, the awareness rate of patients in the observation group on basic knowledge of diseases, medication knowledge, and daily self-care knowledge, medication compliance score, and other health knowledge, as well as self-care abilities such as healthy diet, psychological adjustment, self-care skills, oral care, and perianal care, was significantly higher than that in the control group. Continuous nursing based on the IMB model established scientific and reasonable psychological intervention according to the actual situation of patients to reduce adverse emotions such as anxiety, and we carried out health knowledge promotion for patients to help patients to improve their understanding of the condition, so as to correctly understand the condition, correctly view the condition, and actively cooperate with the nursing work to speed up the recovery of the condition and achieve a good nursing effect. At the same time, we made a home visit to understand the recovery of patients after discharge, so as to solve the existing problems for patients in time, facilitate the next step of nursing plan, and remind patients to seek medical treatment and check-up in time in case of abnormal physical condition during nursing, so as to avoid missing the best treatment time [15, 16].

The article "Analysis of Continuous Nursing Intervention on Aplastic Anemia Patients Based on the “Information-Motivation-Behavioral Skills Model”" was retracted in 2023. Reasons: unreliable results or conclusions; concerns about the data; concerns about the peer review; concerns about the citations.

Although routine nursing intervention has a certain effect of nursing intervention, which can improve the treatment effect and the effectiveness of nursing intervention, it lacks guidance and immediacy, which leads to patients' self-disease control, wrong management cognition, negative emotions, and so on, which seriously affects their physical and mental health. IMB model-based continuous care is a flexible management approach. With the in-depth application and continuous promotion of this nursing method, it has been recognized by more and more people and gradually used in the field of healthcare. As a nursing management method, it has been highly valued by the medical community [17, 18]. IMB-based continuous nursing intervention includes establishing a nursing group, information intervention, motivation intervention, behavior intervention, continuous nursing, and other modules, which are connected with each other to ensure the effectiveness of nursing intervention [19].

Continuous care based on the IMB model improved care satisfaction. It is of great practical significance to find a more reasonable and effective continuous nursing plan in clinic, to enhance the positive feelings of patients and the benefit of disease treatment, so as to improve the clinical prognosis of patients with aplastic anemia and to improve the quality of care for patients with aplastic anemia [20]. The results showed that the nursing quality of life score of the observation group was higher than that of the control group for three months, and the nursing satisfaction of the observation group was significantly higher than that of the control group. In the implementation of IMB-based continuous nursing, nurses give targeted information and motivation intervention to patients, so as to increase the patients' experience of positive emotions. Through nursing care, the bad cognition on diseases was improved, and finally, the patients' satisfaction with nursing care was improved [21].

The article "Analysis of Continuous Nursing Intervention on Aplastic Anemia Patients Based on the “Information-Motivation-Behavioral Skills Model”" was retracted in 2023. Reasons: unreliable results or conclusions; concerns about the data; concerns about the peer review; concerns about the citations.

Continuous nursing intervention based on the IMB model can focus on improving patients' awareness of their own disease-related knowledge, eliminate patients' doubts and anxiety about the disease through face-to-face or online communication, and timely and targeted implement countermeasures for patients' various problems, thus greatly reducing the occurrence of complications [22]. The results showed that the total effective rate of nursing care in the observation group was higher than that in the control group. After the implementation of the IMB-based continuous nursing intervention, through tracking and analyzing the historical data of patients and implementing the contents of health education required by patients, we can make them fully understand the importance of adhering to the treatment. At the same time, adjusting the dosage reasonably according to patients' own physiological conditions can increase patients' tolerance to drugs, reduce their adverse reactions, and then, effectively play a good monitoring role, thus improving patients' compliance with medical drugs and greatly improving the efficiency of nursing.

## 6. Conclusions

IMB-based continuous care can significantly increase the awareness of health knowledge of patients with aplastic anemia, effectively improve medication compliance, significantly enhance self-care ability, and thus, improve the quality of life.

## Figures and Tables

**Figure 1:** Comparison of health knowledge awareness between the two groups. Note: compared with the control group, ^*∗*^*P* < 0.05.

**Figure 2:** Comparison of medication compliance between the two groups. Note: compared with the control group, ^*∗*^*P* < 0.05.

**Figure 3:** Comparison of self-care ability between the two groups. Note: compared with the control group, ^*∗*^*P* < 0.05.

**Figure 4:** Comparison of quality of life between the two groups. Note: compared with discharge, ^*∗*^*P* < 0.05; compared with the control group, ^#^*P* < 0.05.

**Figure 5:** Comparison of nursing satisfaction between the two groups. Note: compared with the control group, ^*∗*^*P* < 0.05.

**Figure 6:** Comparison of the total effective rates of nursing care between the two groups. Note: compared with the control group, ^*∗*^*P* < 0.05.

The article "Analysis of Continuous Nursing Intervention on Aplastic Anemia Patients Based on the “Information-Motivation-Behavioral Skills Model”" was retracted in 2023. Reasons: unreliable results or conclusions; concerns about the data; concerns about the peer review; concerns about the citations.

**Table 1:** Comparison of clinical data between the two groups.

Group	Gender		Age (years)	Degree of education		Routine blood test		
	Male	Female		Up to high school	High school and above	Hemoglobin (g/L)	White blood cells (×10^9^/L)	Platelets (×10^9^/L)
Control group (*n* = 45)	28	17	50.24 ± 5.91	21	24	79.32 ± 18.26	2.94 ± 1.24	68.72 ± 12.07
Observation group (*n* = 45)	26	19	51.07 ± 6.13	20	25	81.52 ± 20.46	3.06 ± 1.51	70.52 ± 11.96
*t/χ* ^*2*^ *value*	0.185		0.654	0.045		0.538	0.514	0.711
*P value*	0.667		0.515	0.832		0.592	0.608	0.479

## Data Availability

The data used and/or analyzed during the current study are available from the corresponding author.
